This article has been retracted.

# Correlation Meta-Analysis of the Efficacy of Inhaled Corticosteroids in Children with Asthma Based on Smart Medical Health

**DOI:** 10.1155/2022/6220774

**Published:** 2022-04-13

**Authors:** Yu Qin, Jing Wang, Jingmin Qin, Ning Yang, Sha Li, Lijia Xu, Yanjun Han

**Affiliations:** ^1^Pediatrics, Xingtai People's Hospital, Zhanjiang 054031, Hebei, China; ^2^Endocrine Department, Xingtai People's Hospital, Zhanjiang 054031, Hebei, China; ^3^Neonatology, Handan Second Hospital, Handan 056001, Hebei, China

## Abstract

Children are the reserve force for national construction, and children's health is now being paid more and more attention. In today's childhood asthma treatment, many are based on the treatment of common cough, and there is no strict division with asthma. Importantly, the efficacy of inhaled corticosteroids in the treatment of childhood asthma has been extensively studied in the medical community. However, there is no clear explanation for its specific efficacy and role. Research on childhood asthma has always been a key topic in medicine. This article aims to conduct a meta-analysis of the correlation between inhaled corticosteroids and asthma in children. This article proposes a more scientific literature screening strategy, which can achieve a higher accuracy rate for meta-analysis. It combines the intelligent medical health system in the analysis of children's asthma to assist in the analysis of curative effects. Such analysis also provides reference significance for related research. The experimental results indicate that inhaled corticosteroids have a good effect on childhood asthma. As the concentration of inhaled glucocorticoid increases, the effect will be better. Specifically, if the concentration is increased by 10%, the effect will be about 15% better, but there are corresponding side effects.

## 1. Introduction

With the advancement of computer information technology, the medical field has increasingly computerized and networked various management forms to reduce costs, facilitate management, and improve the effectiveness of treatment. Early foreign studies have found that the remote management system using telephone, mobile phone text messages, and the Internet as information technology can shorten the distance between the doctor and the patient and help patients adjust their diet and exercise patterns in time. It strengthens blood glucose monitoring and improves the level of disease control. Asthma is a chronic respiratory disease with a high clinical incidence in pediatrics. Although most children can be effectively controlled after effective treatment, there are still some cases of disease that are prolonged and difficult to heal. How to improve the therapeutic effect of asthma is a hot spot in clinical research. Inhaled corticosteroids are the first-line drugs for the treatment of asthma and have definite effects on children with persistent asthma of varying severity. It has been listed as a recommended drug in the global asthma prevention and treatment strategy since 2006.

However, the specific principles and corresponding side effects of inhaled corticosteroids on childhood asthma are not particularly clear. For related studies, more researches are conducted on asthma cases, and there is no comprehensive correlation analysis. Especially with the current technological development of smart medical health, it is very necessary to carry out a correlation analysis of the efficacy of inhaled corticosteroids in children's asthma based on smart medical health.

Therefore, there are two main innovations in this article: (1) In the analysis, it focuses on combining modern smart health medical technology. Based on this, it introduces the application scenarios of smart medical treatment and related technologies. (2) The literature screening strategy in the meta-analysis has been greatly optimized, and some influential and useless factors have been eliminated so that the results of the meta-analysis will be more realistic.

## 2. Related Work

There are different studies on the efficacy of inhaled corticosteroids. Parameswaran K and others believe that there is no consensus on the method of comparing the clinical efficacy of different inhaled corticosteroids. Comparisons need to be made in terms of relative efficacy, and the study should include comparisons of two or three doses. Drug deposition studies and mathematical models of drug pharmacokinetics in the airway can provide supplementary information for clinical drug relative efficacy studies. When estimating the clinical and systemic effects, the fine particle dose and the emitted dose should be considered separately instead of the nominal dose. When comparing with an innovative drug (same compound and same equipment) to evaluate the second entry (generic) drug, if the generic drug meets drug equivalence, it may be appropriate to consider accepting the generic drug as bioequivalence [1]. Qian et al. have studied the side effects of long-term use of inhaled corticosteroids. They believe that these side effects include impaired growth in children, osteoporosis, fractures, glaucoma, cataracts, and thinning of the skin. So they will review the current recommendations on the use of ICS in asthma management to highlight the treatment strategy that strikes the best balance between safety and effectiveness [2]. Hihoriya et al. conducted a randomized and prospective study to determine the efficacy of montelukast as a *β*2 agonist and inhaled corticosteroids in patients with moderate persistent asthma. Experimental results show that montelukast treatment can better improve the clinical symptoms and PFT of patients with moderate persistent asthma [3]. Ema et al. believe that the treatment of the “yellow zone” or worsening of childhood asthma is still controversial. Their goal is to review existing data and consider the effect of increasing the dose of ICS and potential alternatives to this common practice [4]. Hong et al. believe that although nebulized corticosteroids (NebCS) are a key treatment option for young children with asthma or viral wheezing (VIW), there is no uniform recommendation for their best use. The purpose of their study was to clarify the role of NebCSs in the management of acute exacerbations of asthma, asthma maintenance treatment, and VIW treatment in children 5 years of age or younger. The results prove that NebCSs are effective and well-tolerated in the treatment of acute and chronic asthma in patients aged 5 years or younger [5]. Maio et al. believe that dual-agent chemotherapy as the first-line treatment for advanced nonsmall cell lung cancer (NSCLC) is more effective than single-agent chemotherapy. As a second-line treatment, several randomized trials comparing single-drug and dual-drug chemotherapy have been conducted, but each trial is insufficient to detect potential related survival differences. They proved through experiments that dual-agent chemotherapy as a second-line treatment for advanced NSCLC significantly improved the remission rate and progression-free survival. However, it is more toxic than single drugs and cannot improve overall survival [6]. There are also more studies on meta-analysis. Tambini and Roberto conducted a meta-analysis of 5 randomized controlled trials (RCTs) involving 339 patients with acute infectious mononucleosis (IM) treated with acyclovir (ACV). They believe that clinical data does not support the use of ACV for the treatment of acute IM, although the drug has good virological activity [7]. Chu et al. conducted a meta-analysis on suicide and related diseases. Their research conclusion supports the theory of interpersonal relationships: the interaction between frustrated belonging and the perceived burden is significantly related to suicidal ideation. The interaction between frustrated belonging, perceived burden, and suicidal ability is significantly related to more previous suicide attempts. However, the impact of these interactions is moderate. Alternative configurations of theoretical variables are equally useful for predicting suicide risk and theoretically consistent paths. He summarized the limitations and suggestions of interpersonal relationship theory as a framework for understanding the spectrum of suicide [8]. However, there is an obvious deficiency in these theories. That is, modern intelligent medical technology has not been combined and modern medical technology has not been applied, which is not conducive to the combination of technological development and modern medical care. And their research is more on the treatment of asthma, without distinguishing the special group of children. However, this paper pays more attention to the group of children. When conducting meta-analysis, an important point in the search strategy is to limit children. Such strict restrictions on children as research subjects can clearly study the specific effects of inhaled glucocorticoids on children.

The first part of the article introduces the background, significance, and related work of the research on the efficacy of inhaled glucocorticoids in children with asthma and proposes the innovations of this paper. The meta-analysis of childhood asthma and inhaled corticosteroids is proposed, and the intelligent medical treatment based on the Internet of Things is analyzed. The fourth part proposes a meta-analysis of the efficacy correlation and proposes a more scientific literature screening strategy, which can achieve better results. High meta-analysis accuracy: Combined with the intelligent medical health system, it is used to assist the analysis of the curative effect in the analysis of children's asthma, and then the results of the experimental part are analyzed and summarized.

## 3. Introduction of Smart Medical and Health Related Technologies

### 3.1. Childhood Asthma and Inhaled Corticosteroids

Childhood asthma seriously harms children's health worldwide. For many years, it has become the most common public health problem in childhood [9]. The incidence and mortality of bronchial asthma in children are on the rise worldwide. Through in-depth investigation and clinical research analysis among clinical workers in many countries and regions, it has been found that the prevalence of bronchial asthma in children has increased significantly in the past 10 years. The incidence and prevalence of asthma in the world have also increased substantially [10]. In recent years, the prevalence of bronchial asthma in children in China has gradually increased. There are currently about 20 million asthma patients in China. In 1996, the domestic pediatric bronchial asthma investigation team conducted a survey of normal and ill children aged 6–12 years in various provinces, regions, and counties in China. The results found that the incidence of bronchial asthma in children in China has increased significantly compared with the previous period. By the end of 2010, the results of the survey of childhood asthma (6–12) in existing cities in China showed that the incidence of asthma was 0.25%–4.63%, with an average of 1.97%. The results of the reinvestigation in 2006 were 0.35%–4.38%, an average of 2.34%, and an average increase of 74.84% over the past 10 years. Among them, Shanghai is 5.24%, currently ranking first in the country [11, 12]. As humans continue to transform and pollute the Earth, a series of changes will occur in the current atmospheric environment, biological species and ecology, and dietary structure. Therefore, allergic symptoms and bronchial asthma will gradually show an upward trend. Asthma is mainly composed of a variety of inflammatory cells and cellular components that participate in the onset and pathological evolution of asthma. The main clinical manifestations of patients have increased airway responsiveness and recurrent wheezing, shortness of breath, chest tightness, and (or) coughing. At present, inhaled corticosteroids are the most effective anti-inflammatory drugs for the first-line treatment of asthma. It mainly reduces the chronic inflammation of the airway by reducing the activation of T lymphocytes and inhibiting the production of cell-related inflammatory factors [13]. Helper T lymphocytes also play an important role in immunity and regulation in chronic airway inflammation in children with asthma [14].

With the in-depth clinical understanding of the pathogenesis of asthma, people have gradually gained new understanding and research on the mechanism of action of glucocorticoids [15]. Through long-term inhalation of glucocorticoids to understand the pathological and related physiological changes of children, it is helpful to clarify the influence of glucocorticoids on the intrinsic immune function of children. It can provide a reliable basis for the Formulation of glucocorticoid medication regimens in clinical research and the in-depth study of the specific mechanism of glucocorticoids [16]. A large amount of literature analysis pointed out that IgE, TNF-*α*, IL-8, IL-17, LTB4, and other inflammatory factors played an important role in the occurrence, development, and evolution of asthma. Therefore, glucocorticoid anti-inflammatory therapy is an important part of the treatment of asthma. In reality, we mainly use inhaled corticosteroids to treat asthma in clinical practice, which has a definite effect [17]. Therefore, studying the related pathogenesis and new treatments of bronchial asthma has become a global health problem to be solved. Therefore, we should pay enough attention and work hard to solve it from now on. Active and reasonable detection of children with bronchial asthma can prompt the survival and comfort of the children, improve the symptoms and duration of asthma attacks, and reduce the economic burden of children with children [18].

### 3.2. Meta-Analysis

There are two main schools of statistics: the classical frequency statistics school and the Bayesian school scholars have contributed to the development of network meta-analysis (NMA). And some scholars have compared the application of the two faction theories in meta-analysis [19]. The frequency school's NMA method is based on the assumption that the effect scale obeys normal distribution. Bayesian statistics takes the target parameter *θ* as a random variable with a priori distribution. After obtaining the sample information, it obtains comprehensive information about the posterior distribution *π*(*θ*|*x*) of *θ* through simulation iteration so as to obtain the Bayesian estimation of the parameter *θ*. In recent years, it is based on the Bayesian NMA viewpoint put forward by Higgins and Whitehead. Many scholars have gradually developed multiple models such as simple Bayesian NMA, NMA under the framework of generalized linear models, and multilevel hierarchical Bayesian NMA, collectively referred to as “Bayesian NMA model” [20]. The following is an introduction to the NMA model algorithm based on Bayesian model averaging.

The symbol *β* represents the parameter vector to be estimated, and *N*_*k*_ represents the *k*-th model in the better model space. Let A denote the observed data sample, the posterior density distribution of *β* can be written in the following form:

(1) $$\begin{array}{c} P\left(\beta |A\right)=\sum_{K-1}^{K}P\left(\beta |A,N_{K}\right)P\left(N_{K}|A\right). \end{array}$$

In formula (1), *A* represents a set of *i* samples. According to formula (1), the estimated value and variance of the parameter vector *β* to be solved are as follows:

(2) $$\begin{array}{c} E\left(\beta |A\right)=\int_{-\infty }^{+\infty }\beta \left[\sum_{K-1}^{K}P\left(\beta |A,N_{K}\right)P\left(N_{K}|A\right)\right]d\beta , \end{array}$$

(3) $$\begin{array}{c} Var\left(\beta |A\right)=\int_{-\infty }^{+\infty }{\left[\beta -E\left(\beta |A\right)\right]}^{2}\left[\sum_{K-1}^{K}P\left(\beta |A,N_{K}\right)P\left(N_{K}|A\right)\right]d\beta , \end{array}$$

or abbreviated as follows:

(4) $$\begin{array}{c} E\left(\beta |A\right)=\hat{\beta }P\left(N_{K}|A\right), \end{array}$$

(5) $$\begin{array}{c} \text{Var}\left(\beta |A\right)=V1+V2. \end{array}$$

In formula (5), *V*1 is the error between models, and *V*2 is the error within the models, expressed as follows:

(6) $$\begin{array}{c} V1={\sum_{K-1}^{K}P\left(N_{K}|A\right)\left(\hat{\beta }-\sum_{K-1}^{K}P\left(N_{K}|A\right)\hat{\beta }\right)}^{2}, \end{array}$$

(7) $$\begin{array}{c} V2=\sum_{K-1}^{K}P\left(N_{K}|A\right)Var^{2}\left(\beta |A,N_{K}\right). \end{array}$$

It can be seen from the introduction that determining the posterior probability of the model is the key to the model. The parameter conditions make the model optimal. Then the posterior probability is as follows:

(8) $$\begin{array}{c} P\left(\Delta |N_{K},A\right)=\int P\left(\Delta |\beta_{K},N_{K},A\right)P\left(\beta_{K}|N_{K},A\right)d_{\beta }. \end{array}$$

In formula (8), (1, 2, ..., *k*) is the unique regression parameter vector of the better model *N*_*k*_. Use maximum likelihood estimation to approximate as follows:

(9) PΔ|NK,A≈PΔ|NK,β^,K A.

This estimate can be used as a very good approximation when it is considered uncertain about the model in subsequent proofs, and it is used by subsequent scholars [21, 22].

Write the model's posterior probability estimate (BIC) as a Bayesian Formula, as shown in the following formula:

(10) $$\begin{array}{c} P\left(N_{K}|A\right)=\frac{P\left(A|N_{K}\right)P\left(N_{K}\right)}{\sum_{J=1}^{K}P\left(A|N_{K}\right)P\left(N_{K}\right)}, \end{array}$$

In formula (10), *P*(*N*_*k*_) is the prior probability of model *N*_*k*_, so formula (10) can be written as follows:

(11) $$\begin{array}{c} P\left(N_{K}|A\right)=\frac{P\left(A|N_{K}\right)}{\sum_{J=1}^{K}P\left(A|N_{K}\right)}. \end{array}$$

In formula (11), *P*(*A* |*N*_*k*_) can be written in the form of a marginal likelihood function, that is,

(12) $$\begin{array}{c} P\left(A|N_{K}\right)=\int P\left(A|\beta_{K},N_{K}\right)P\left(\beta_{K}|N_{K}\right)d\beta_{k}. \end{array}$$

The estimated value of formula (12) is obtained by the Laplace approximation method as shown in the following formula [23]:

(13) $$\begin{array}{c} \log\left(P\left(A|N_{K}\right)\right)=\log\left(P\left(A|\beta ,N_{K}\right)\right)-\left(\frac{d_{k}}{2}\right)\log\;n+o\left(1\right). \end{array}$$

*Kd* in formula (13) represents the number of parameters to be estimated in the *k*-th model *N*_*k*_, and *n* represents the number of samples. The Bayesian information criterion is as follows:

(14) $$\begin{array}{c} BIC_{K}=-2\;\log\left(P\left(A|N_{K},\beta_{K}\right)\right)+d_{k}\log\;n. \end{array}$$

It is further transformed into the following formula:

(15) $$\begin{array}{c} -\frac{BIC_{K}}{2}=\log\left(P\left(A|N_{K},\beta_{K}\right)\right)-\left(\frac{d_{k}}{2}\right)\log\;n. \end{array}$$

Therefore, the posterior probability expression of the BIC model is as shown in thefollowing formula:

(16) $$\begin{array}{c} P\left(N_{K}|A\right)=\frac{\exp\left(-BIC_{K}/2\right)}{\sum_{J=1}^{K}\exp\left(-BIC_{K}/2\right)}. \end{array}$$

So far, the NMA model algorithm based on Bayesian model averaging has been introduced. The uncertainty of models and parameters and the comprehensive and effective use of information are the main factors that affect the results of meta-analysis. This paper uses the Bayesian Model Average (BMA) method to model and optimize the meta-analysis and integrates the information of the alternative models and variables to control the uncertainty of the model and effectively utilize the rich key information.

### 3.3. Smart Healthcare

The application of advanced technology in medical testing instruments provides favorable conditions for the effective diagnosis of public pathology, which can fully meet the needs of medical diagnosis [24]. However, the medical testing instruments currently used in the market are usually bulky and expensive. When in use, it needs to be in close contact with the test object, and the test object cannot move casually. It is generally not suitable for monitoring a large range of high-risk infectious disease patients, and it is not suitable for patient populations that are geographically dispersed but require real-time monitoring [25]. Therefore, through heterogeneous wireless network coordination, a seamless connection between WLAN and mobile communication network is realized in a ubiquitous network environment, which is conducive to the health prevention and control center to grasp the information of the monitored patient at any time and any place. Thus, it provides a strong basis for the adoption of effective diagnosis and treatment plans, which is very feasible and has national strategic application value for preventing and controlling the spread of sudden major infectious diseases.

However, due to the characteristics of China's national conditions, it is difficult to use the network for remote management. The development of medical technology in the new era is rapidly developed in conjunction with the development of other information technologies [26]. In modern medicine, digital, visual information, high-precision sensors, electromagnetic imaging, and other technologies are used to make it more convenient to observe various information of the human body. It makes the diagnosis more accurate, and people can get better medical services. Before the advent of these technical devices, doctors could only obtain the physiological state of patients by means of experience and hearing. This method relies more on the subjective ability of the doctor and has a great risk. At the same time, the technology is difficult to promote among new doctors [27]. Therefore, the medical diagnosis technology at that time mainly relied on the doctor diagnosed. With the development of electronic information, people have discovered that electromagnetic waves, sound waves, and other information can be used to realize the manifestation of human physiological signals. As a result, the medical diagnosis will no longer rely on the doctor's experience but use high-tech to accurately reflect the physiological changes of the human body [28]. Among them, the application scenarios of smart medical systems can be divided into isolated areas and nonisolated areas, as shown in Figure 1:

As shown in Figure 1, the descriptions of the two scenarios are as follows.

Scenario 1: When a patient is isolated in a designated place, the portable multiphysiological parameter collection terminal will be connected to the wireless AP point in the environment through WiFi. Since the patient is at the isolation point, it is not convenient for medical staff to enter and observe the patient's condition at any time, so it must be linked through the device. However, the network of isolation points needs to be relatively stable to meet the needs of medical staff and patients. For example, in the case of a pneumonia epidemic, the patient is in the isolation room, and all data are tested by wearable devices.

In these two scenarios, a large-scale high-speed mobile network and a small-scale low-power wireless access technology can be organically combined. It realizes the monitoring of infectious epidemics in the two scenarios and ensures a seamless connection in two scenarios. Monitoring personnel can use mobile phones, laptops, and other terminal devices to access the application server of the Health Prevention and Control Center through the Internet, regardless of whether they are working in the quarantine area or when they are outside the quarantine area. It knows the physiological parameters of the monitored object in time so as to make corresponding prevention and control measures.

Among them, its specific architecture and services are shown in Figure 2:

Intelligent medical platforms based on the Internet of Things include cloud computing centers, hospital platforms, home terminals, service centers, etc. As shown in Figure 2, the monitoring system is divided into 4 layers, which are the monitoring terminal, information interaction system, database, and monitoring center. For the monitoring terminal, it is targeted at specific patients. They obtain basic information through their own or hospital-provided testing equipment, or the equipment can take and upload it by themselves. This is very convenient for the patient and for the nurse, the simple and time-consuming measurement operation is avoided, and the patient can solve it by himself. For the second-level information interaction system, the network, data processor, data collector, etc., are integrated to achieve the functions of uploading and data processing. The data collected by patients is simply classified and analyzed through the information interaction system, and simple statistical processing is performed to form a report directly to the doctor and upload the data to the third-tier hospital's database so that it is more convenient for doctors to make accurate judgments about the patient's overall situation and recent conditions. For the fourth layer, it is aimed at medical staff. They use the testing center to conduct unified testing on patients, and they can respond to the situation as soon as possible. It accurately locates the data of the problem, which is the location where the problem occurs, so that the targeted and timely treatment can be carried out.

## 4. Meta-Analysis of the Correlation of Curative Effect

### 4.1. Literature Inclusion Strategy

The inclusion and exclusion of the literature should follow practical principles, and there should be information about the efficacy of inhaled corticosteroids in children. Specifically, the following strategies:

1. Literature inclusion criteria
2. The original documents are observational studies (cohort studies, cross-sectional studies, time series, and case crossover);
3. It studied the efficacy of inhalable glucocorticoids;
4. The research object is children, and the diagnostic criteria or methods of asthma are described in the literature;
5. The results of the analysis of the curative effect on asthma are reported in the literature;
6. For the repetitive literature, choose the one with the closest topic to this one;
7. The languages are limited to Chinese and English.
8. Document exclusion criteria
9. News, letters, summaries, reviews, abstracts, and lectures, etc.;
10. It does not describe the diagnostic criteria or methods of childhood asthma;
11. Incomplete and unavailable documents provided by the data;
12. The literature research population includes adults and children, but children's data cannot be extracted separately.
13. Publication languages are other than English and Chinese.
14. Literature search strategy
15. Documents were screened by computer and searched in the research papers databases of HowNet, Wanfang, and Zhangqiao.

The time is set from 2016 to present, and the papers are roughly screened based on the keywords of the papers, and then the initially selected documents are manually screened. The specific screening steps are shown in Figure 3.

As shown in Figure 3, the first step is to search through keywords and a total of 5,324 papers were screened, and after deleting duplicates, 3491 papers remain. Then the literature was screened according to the principle of exclusion, leaving 189 articles, and after screening the full text, 31 articles remained, and then 31 articles were meta-analyzed.

Among them, the 31 articles after screening are classified, and the country classification is shown in Table 1; the research category is shown in Table 2. Among the 31 documents in Table 1, there are 13 in the United States, 9 in China, 6 in Germany, and 3 in Japan. In Table 2, there are 11 studies for cohort studies, 13 for cross-sectional studies, 7 for case crossover studies, 3 for time series studies, and 19 for inhaled corticosteroids.

### 4.2. Meta Analysis Results

1. The quality of the articles after screening is shown in Figure 4.
2. In Figure 4, based on the degree of suitability between the research content of the literature and this article, the literature quality of the four countries is shown in the figure. It can be found that in the four countries, the quality of the literature is relatively high, with more than 25% of the articles of excellent quality. Among them, because there are only 3 Japanese documents, the excellent rate reached 66.6%. Therefore, the extraction of the literature is quite satisfactory.
3. Meta result analysis
4. Thirty-one articles have studied the effect of inhalable corticosteroids on childhood asthma. There is a certain degree of bias in the literature. This paper chooses the random-effects model to merge the results. The results of the meta-analysis are shown in Figure 5. It can be seen in the figure that most of the studies are single studies with a large confidence interval. The diamond is on the vertical line, indicating that there is no difference between the two groups.
5. Heterogeneity
6. The heterogeneity analysis of the included 31 articles was carried out, and a funnel chart was drawn for them, as shown in Figure 6.
7. In Figure 6, the ordinate represents the error. The abscissa is the odds ratio (OR). It can be seen from the figure that most of the points are concentrated at the top, and some points are scattered at the bottom. This shows that most of the samples are large samples, and only a few small samples are scattered at the bottom. For the funnel graph, there are missing corners in the graph, which indicates that the sample has publication bias, and there are two points outside the funnel. For the 95% confidence interval, this means that there is no obvious heterogeneity between the research samples.
8. Publication bias
9. Egger's linear regression method is used for the publication bias test because this method can take into account the existence of the intercept term. As shown in Figure 7, it can be found from the regression graph that the sample points have a downward trend in the graph, and the fitted trend line is also downward. This woman shows that there is a publication bias in the effect of inhalable corticosteroids on asthma. This is the same as the result of the funnel chart in Figure 6, and there is publication bias. It is more obvious that the sample has publication bias because there is a certain bias in the selection of the literature.
10. Sensitivity analysis
11. Finally, a sensitivity analysis of the literature is carried out, and we adopt the method of exclusion one by one to carry out the sensitivity analysis. As shown in Figure 8, the results show that no single article can significantly affect the overall heterogeneity. A sensitivity analysis was performed on the results of the overall combined analysis using the one-by-one elimination method. That is, each study was excluded. Meta-analysis was performed again on the remaining studies, and the results showed that the sensitivity analysis results did not change significantly compared with those before the exclusion. The credible interval of each indicator overlaps with the original value to a large extent, suggesting that the results of the meta-analysis of this study are more reliable.

### 4.3. Efficacy Analysis

The experimental data is an existing data sample in the hospital, which is analyzed on statistical software. To explore the clinical efficacy of NIPPV (noninvasive positive pressure ventilation) in the treatment of bronchial asthma. A total of 162 patients with bronchial asthma who were admitted to a hospital from June 2014 to May 2018 were included in the study, and the clinical efficacy and symptom disappearance time of the control group (conventional treatment) and the observation group (inhaled glucocorticoid treatment) were compared.

1. The efficacy of inhaled glucocorticoids
2. From Figure 9, we can see that inhaled corticosteroids have a relatively good effect on childhood asthma. When *F* ≥ 2, the effect can be at a relatively high value. The highest point can reach 0.98.
3. Diagnosis and treatment accuracy
4. As can be seen from Figure 10, the accuracy of inhalable corticosteroids for the diagnosis of asthma is also relatively high. The accuracy of diagnosis can reach more than 90% at different concentrations, and with the increase of time, the accuracy of diagnosis and treatment will become higher and higher.

## 5. Discussion

Childhood asthma is a source of greater harm to children's health and may cause irreversible damage to lung damage. At present, there are also some medicines for treating children's asthma, and there are many treatment methods. However, there are still relatively few treatments for radical cures or no side effects. After all, children are in a poor physique. Corresponding body functions have not yet been fully perfected. Too much medicine or adult medicine is not reasonable. This article refers to the research of other scholars and adopts the method of meta-analysis. The 31 documents included in the meta-analysis are all observational studies. Among them, there are 11 cohort studies, which are a type of research design with better etiology, and the overall sample size of the included literature is relatively large. The cohort studies and case crossover studies included in this article use the NOS score to assess the risk of bias. Of the 18 articles, 12 have a score greater than or equal to 8. The included cross-sectional studies were evaluated using the AHQR scale, and the coincidence rates of 9 items were all high. The quality of the literature entered into this analysis is relatively high, and there is a dose-effect relationship between acute and chronic effects. There is a certain degree of clinical heterogeneity in the literature included in this article, such as different regions and different age groups. Therefore, a further subgroup analysis of inhalable glucocorticoids is still not possible to completely eliminate the heterogeneity in the literature. At the same time, the chronic effect literature has obvious publication bias. Combined with the GRADE evidence quality evaluation tool, the quality of evidence for the efficacy of inhaled glucocorticoids on childhood asthma is relatively high. However, the principle of its side effects is still not clear enough, and some related studies believe that it will affect the height development of children. Therefore, the efficacy of inhaled glucocorticoids remains to be analyzed.

However, the limitations of this study are as follows: (1) The quality of the included RCTs (Used to evaluate the possibility of bias) is not the same. Although they all have the quality that can be included, high-quality, high-level RCTs are more important in future studies. In future research, the grouping information and methods, as well as the situation of loss to follow-up and withdrawal, should be described in detail. (2) There must be heterogeneity between different studies, which will have a certain impact on the results of meta-analysis. These may be caused by different basic conditions, such as age, gender, and disease course. Moreover, the different types and doses of oral drugs in the control group may also affect the results. (3) The existence of publication bias is always a problem, and differences in research results and sample size can affect publication bias. This may be related to negative results. That is, articles that do not have any significant differences in results are more difficult to publish. (4) The research on smart medical technology has not fully targeted children's asthma. The literature is not deep enough for its research, which means that the article has not fully used the smart medical technology of children's asthma.

## 6. Conclusions

This study systematically evaluated the efficacy of inhalable glucocorticoids on children with asthma and preliminarily summarized its laws in the various research literature, with a meta-analysis as a result. When the two are not affected by the prevalence, the value range is between (0, 1), and the closer to 1, the higher the diagnostic accuracy of the experiment to be evaluated. In addition, as the pathological stage increases, the sensitivity and specificity values gradually increase. This indicates that the efficacy of inhalable glucocorticoids increases with the increase in concentration, and the misdiagnosis rate gradually decreases. The article also emphatically mentioned the application of smart medicine and analyzed its structure and application. It is hoped that smart medical technology can be applied to the case study of childhood asthma in the follow-up research, and combined with the technology of the system platform, to deeply explore the curative effect and influence of inhaled corticosteroids on childhood asthma.

## Figures and Tables

**Figure 1:** Application scenario diagram of the intelligent medical real-time monitoring system.

**Figure 2:** The functional block diagram of the intelligent medical real-time monitoring system.

**Figure 3:** Screening steps diagram.

**Figure 4:** Document quality evaluation chart.

**Figure 5:** The relative risk diagram of the efficacy of inhalable glucocorticoids.

**Figure 6:** OR funnel chart.

**Figure 7:** Regression graph of the effect of inhalable glucocorticoids on childhood asthma.

**Figure 8:** Sensitivity analysis graph.

**Figure 9:** Fibroscan diagnosis *F* ≥ 2.

**Figure 10:** Three SROC curve of sCD14-ST diagnosis accuracy of asthma.

**Table 1:** Document country list.

Country	Number of documents	Percentage (%)
America	13	41.9
China	9	29.0
Germany	6	19.4
Japan	3	9.7

**Table 2:** Literature research category table.

Research category	Number of documents	Percentage (%)
Array research	11	20.8
Cross-sectional study	13	24.5
Case crossover study	7	13.2
Time series research	3	5.7
Inhaled glucocorticoid research	19	35.8

## Data Availability

No data were used to support this study.
